# Four-Way Evolutionary Game Analysis of Government Project Bidding Collusion in a State of Limited Rationality Based on Prospect Theory

**DOI:** 10.1155/2022/6092802

**Published:** 2022-01-21

**Authors:** Chongsen Ma, Yun Chen, Sirui Nie

**Affiliations:** College of Transportation Engineering, Changsha University of Science and Technology, Changsha, Hu Nan 410000, China

## Abstract

Controlling collusion in government bidding is a prerequisite for ensuring social justice and the smooth operation of projects. Based on the prospect theory, this article establishes a four-party evolutionary game model for tenderers, enterprises with higher willingness to collude, enterprises with lower willingness to collude, and supervising enterprises. The study uses replication dynamics to analyze the stability of strategy selection after the evolutionary game. The results show that higher project base returns increase the probability of collusion, while lower market competition, higher risk aversion, and stronger collusive regulation all reduce the probability of collusion. When regulators adopt a strong regulatory strategy, the remaining project participants tend to choose a noncollusive strategy.

## 1. Introduction

Tendering is an effective way of acquiring and allocating resources developed over time in social and economic activities [1]. China's government investment projects primarily use bidding to determine the project builder. However, due to the asymmetry of information between the bidding parties, the trend of interests, and the imperfection of the restraint mechanism, the parties involved in the bidding process will produce collusion and other illegal and irregular behaviors to maximize their interests [2]. These behaviors will seriously affect the orderly development of China's construction market; therefore, it is of great theoretical and practical significance to control collusion in government investment projects' bidding processes.

The principal-agent theory and game theory are the main methods used by domestic scholars to analyze the engineering collusion phenomenon. Xie points out that although excessive competitive pressure in the construction market can induce collusion, its root cause is excessive returns and insufficient punishment [3]. According to Yu, information asymmetry caused by multiple entrustment relationships in government-invested construction projects and the low cost of collusion are the main reasons for its emergence [4]. Cheng et al. argue that high profits in engineering projects' bidding processes are the leading cause of vertical collusion [5]. Miklos-Thal argues that collusion is possible without additional costs, but the presence of additional costs can facilitate its occurrence in cases of asymmetric collusion costs [6]. Through their investigation, Yun Chen et al. found that technical and environmental causes are more critical to creating vertical collusion [1].

Current research provides diverse solutions on control measures for collusion in bidding in government investment projects. For example, Wu et al. combined prospect theory and game theory to establish a collusion regulation deterrence model to regulate collusion in government investment projects [7]. Wang Xianjia et al. constructed a control model to prevent collusion between bidding agents and tenderers in the bidding process based on the “prisoner's dilemma” game [8]. Chen et al. used the cooperative game model to analyze the conditions of collusion and provide a reference for the policy formulation of collusion control [9]. Zhang and Wang constructed a two-sided game model between owners and bid evaluation experts and established a control model to prevent collusion with bid evaluation experts [10].

The above literature review shows that although more scholars have researched vertical collusion in government investment project bidding, the research results have certain limitations due to the methods adopted, mainly focusing on game theory and principal-agent theory. The existing studies focus less on each participant's risk attitude and propensity on a behavioral decision. For simplification, the existing game models on the game behavior research process of vertical collusion process usually consider only two-party or three-party games, which cannot entirely reflect the actual situation [11–21]. In the bidding process of government investment projects, each participant shows different degrees of risk awareness and risk appetite due to different risk management behaviors in the face of complex and variable risk factors. The dynamic formation process of owners' and contractors' risk management behaviors can be seen as the process of both parties adjusting their strategies to form a final stable strategy through trial and error, summarization, and imitation. These methods are consistent with the characteristics of evolutionary games and can be analyzed by evolutionary game theory. This study helps each participant in the bidding process of government investment projects make reasonable risk management decisions by examining each participant's evolutionary behavior in the bidding process of government investment projects. The value function of prospect theory is introduced into the evolutionary game theory, based on the consideration of different collusion tendencies. The risk-benefit perception matrix is constructed to analyze the evolutionary process and inner law of the decision-making behaviors of bidding parties, subjects with high collusion tendencies, subjects with low collusion tendencies, and regulators. Based on MATLAB simulation, the influence of relevant factors on the evolutionary results is analyzed. Therefore, this article introduces prospect theory based on the original evolutionary game approach to analyze collusion in the bidding process. This article divides the bidders into high collusion willingness bidders and low collusion willingness bidders for analysis so that the model is more suitable to the actual situation.

The innovations of this paper are mainly in two ways:

1. Most of the existing studies related to evolutionary games use two-party or three-party games, regardless of the topic and context of the paper's research. This study considers the game behaviour of four parties in the process of vertical collusive control of government investment project bidding. It has certain contribution in the model approach and broadens the existing research ideas and research perspectives.
2. In the current research on vertical collusion in bidding for government investment projects in China, most of the parameters for the benefits and costs of each entity are set only considering the impact of penalties such as fines and penalties. Less consideration has been given to social recognition and the possible impact on future development gains. The study introduces indicators such as the degree of market competition and loss of social recognition to provide an in-depth analysis of the benefits and costs of each subject. By diversifying the parameter model and introducing more detailed considerations, the results of the study are more relevant and reliable.

## 2. Simulation Model Construction

### 2.1. Simulation Analysis Model for the Evolution of Collusive Bidding Behavior

Vertical collusion is repeatedly prohibited in the bidding process of government investment projects. Existing studies usually view bidders as a whole, and they are considered to have a high degree of similarity in their behavior. However, in practice, different bid groups have different perceptions of factors such as potential benefits, penalties, and the probability of detection of vertical collusion, as well as large differences in the business philosophies of different companies. Even under the same external conditions, there are significant gaps in decision making between different bid groups. Therefore, this article divides bidders into two groups, high and low, according to their willingness to participate in collusion to improve the study's credibility. Bidders with high collusion willingness will actively seek collusion opportunities and promote collusive behavior. Firms with low collusion willingness are less likely to collude when faced with opportunities, and at the same time, may report collusive behavior.

In this study's evolutionary game-theoretical model, there are four game subjects: bidders, enterprises with a high willingness to collude, enterprises with a low willingness to collude, and regulators. The four parties influence each other in the bidding process. Some enterprises may choose to collude with the government to obtain a project, adopting forms such as bid-rigging and bid-rigging to obtain excessive profits; the regulator (including the regulator and the people) accepts the government's commission or spontaneously carries out supervision of the project. The government entrusts the regulators (including the regulator and the people), or they spontaneously supervise the project; the regulators' management also has a certain influence on the behavior of the government and enterprises. This article focuses on the vertical collusion in the bidding process of government investment projects. In government investment projects, the government side is the bidding side. In the bidding process, there is a bidding side to release the project; enterprises obtain the project by bidding. However, the bidding process involves inconsistency of different enterprises' business philosophies and decision-making tendencies. As such, enterprises with higher willingness to collude and those with lower willingness to collude will have a higher possibility of providing benefits to the bidders and seeking the opportunity to collude to obtain the project. Companies with a lower willingness to collude will not actively seek opportunities for collusion and will monitor and report any collusion found. Bidders, companies with a high willingness to collude, and companies with a low willingness to collude are all subject to the regulator's supervision. Due to the incomplete symmetry of information and the imperfect rationality of the government and the parties involved in the game, all parties involved may act opportunistically in the project's construction process, making it impossible for all parties to obtain maximum utility.  Figure 1 shows the relationship between the various interest subjects in the bidding process.

### 2.2. Model Assumptions

**Assumption 1 .**

The four main players in the game are the bidders, enterprises with higher willingness to collude, enterprises with lower willingness to collude, and the regulator. In the bidding process, the bidders prefer enterprises involved in collusion as the winning bidders. The colluding enterprises must pay a certain extra cost while fulfilling the contract conditions. The regulators monitor the enterprises involved in bidding to reduce corruption and collusion in the project. The enterprises not involved in collusion have a certain probability of reporting parties involved in collusion to ensure their rights and interests.

**Assumption 2 .**

In the project bidding process, all stakeholders are finite rational “economic agents,” i.e., the parties involved in the project are not fully rational. In the game process, all four parties play a limited number of repeated games.

**Assumption 3 .**

Traditional evolutionary games are based on expected utility theory. They do not consider the influence of the various project participants in the decision-making process on the game's outcome due to psychological perception factors. This article addresses the problem by using the prospect theory proposed by Kahneman et al. to modify decision-makers' inconsistent risk preference behavior. The theory states that one cannot have an absolute perception of losses and gains but rather a relative value of perceived losses, expressed using ∆*ω*1, the difference between the actual loss or gain *ω*1 and a reference point *ω*0. This reference point is subject to the influence of the decision-maker and is chosen differently across research areas. This paper chooses 0 as the reference point. In prospect theory, the expected total utility of a decision is measured using the value function *v* (∆*ω*1) and the weighting function *p*. The prospect value is

(1) $$\begin{array}{c} V=\sum_{\iota }\pi \left(p\iota \right)v\left(\Delta \omega \iota \right). \end{array}$$

Each participating subject makes a judgment on its next move based on its perceived value of the lost gain, and the value function is

(2) $$\begin{array}{c} V\left(\Delta \omega_{i}\right)\;=\left\{\begin{array}{cc} {\left(\Delta \omega_{i}\right)}^{\theta }, & \Delta \omega_{i}\geq 0,\\ -\lambda {\left(-\Delta \omega_{i}\right)}^{\theta } & \Delta \omega_{i}<0, \end{array}\right)\; \end{array}$$

where *θ* is the risk attitude coefficient, indicating the game subject's marginal degree of diminishing perceived value of profit and loss. *λ* is the loss avoidance coefficient, indicating the game subject's sensitivity to loss; the larger the value, the greater the game subject's sensitivity to loss. At the same time, the game subject judges the weights according to the actual situation of the event, using the formula:

(3) $$\begin{array}{c} \pi \left(p_{i}\right)\;=\;\frac{p^{\gamma }}{{\left(p^{\gamma }+{\left(1-p\right)}^{\gamma }\right)}^{1/\gamma }}. \end{array}$$

Except for minimal probability events, *π*(*p*_*i*_) < *p*_*i*_, *π*(*p*_*i*_)+*π*(1 − *p*_*i*_) ≤ 1 and *π*(1) = 1, *π*(0)  = 0. In prospect theory, the probability of a low-probability event occurring is usually overestimated, and the probability of a high-probability event occurring is usually underestimated.

**Assumption 4 .**

The government has two strategies based on its interests and overall interests: participating in government-enterprise collusion or not participating in government-enterprise collusion. Similarly, enterprises with a high willingness to collude have two strategies: to participate in collusion actively or not actively participating in collusion. Enterprises with a low willingness to collude can either report collusion or not. Regulators also have two strategies: to strongly or weakly regulate collusion. A tenderer's probability of adopting a government-enterprise collusion strategy is *x*. The probability of a firm with a high collusion willingness implementing an active collusion strategy is *y*, the probability of a company with a low willingness to collude adopting a reporting collusion strategy is *z*, and the probability of a regulator adopting a strong regulatory model is *m* (0 ≤ *x* ≤ 1, 0 ≤ *y* ≤ 1, 0 ≤ *z* ≤ 1, 0 ≤ *m* ≤ 1). Thus, the tenderer's probability of not participating in government-business collusion is 1 − *x*. The probability of companies with high willingness to collude of not actively participating in collusion is 1 − *y*, the probability of companies with low willingness to collude of not reporting collusion is 1 − *z*, and the probability of regulators adopting the weak regulatory model is 1 − *m*.

**Assumption 5 .**

The government's choice to engage in collusion means that, in the bidding process, it will give preference to a company willing to collude as the winning bidder; if it chooses not to collude, the government will choose the best company as the winning bidder. Selecting a company with a high willingness to collude means that the company will actively seek collusion plans from the authorities, including bribes, etc., to obtain the project. Choosing not to participate in collusion actively means that, although the enterprise is willing to collude, it does not want to pay extra for collusion. Enterprises with a low willingness to collude that choose to report collusion indicate that this type of enterprise will inevitably report any discovered act for higher authorities to handle. The regulator's choice of a strong regulatory model for collusion can be costly, but collusion will be detected in all regulated projects. The choice of a weak regulatory model means that collusion in regulated projects will potentially go unnoticed.

### 2.3. Parameter Setting and Model Construction

Suppose the government chooses to participate in the collusion with an enterprise. In that case, it will receive the social benefits of completing the project. However, it still has to bear the loss *R*_1_ for the nonconformity of the capacity of the vertically colluding enterprise, with a probability of *α*. The probability of society discovering the collusion is *β*, and the loss of *S*_1_ (including market distortion and the collusion will cause loss of trust, etc.). The government will receive the basic benefits of the completed project *F* regardless of whether it is involved in collusion. Still, because no corrupt practices occur during the project bidding process, the sociopolitical climate will increase along with people's trust in the government, with a gain of *F*_2_.

The probability that a firm with a higher willingness to collude will choose to participate in the collusion strategy is *β*. The project's supply affects the probability that a firm with a higher willingness to collude will choose the collusion strategy. The degree of market competition affects SS, the more intense the competition, the higher the probability of choosing collusion and the higher SS. Suppose firms with a higher willingness to collude decide not to participate in collusion. In that case, the probability of their bid actively is reduced to *R*_3_ while simultaneously reducing the possibility of firm expansion, bringing a loss of *S*_5_.

A firm with a low willingness to collude chooses the strategy of reporting on collusion, in which case the gain is 0; there is a risk of resistance from the government and colluding firms, bringing a loss of *S*_6_, but increased social recognition represented by *F*_4_. The probability of the report being discovered by the government and colluding firms is *D*; choosing not to report on collusion yields an additional gain of *F*_5_.

The supervising enterprise gains *F*_6_ regardless of which model it chooses. Choosing to select a strong supervision model brings an increase in recognition, represented by *F*_7_, but may be subject to hostility from the regulators involved in the collusion, bringing losses of *S*_6_. Suppose the supervising enterprise does not collude with the enterprise and the bidder in the strong supervision model, choosing the weak supervision model gives a fixed gain of *F*_6_, while there is a probability of *G* that the enterprise will choose to collude with the contractor. The firm has a *G* probability colluding with the offerer, which provides an additional *F*_7_ gain (including the potential gain from more opportunities for cooperation between the offerer and the firm) and a *D* probability of being discovered, resulting in an *S*_7_ loss.

The parameters and their explanations are shown in Table 1.

According to prospect theory, the decision-making group develops perceived utility when facing uncertain costs and benefits. This article assumes that the cost of expenditure and the legitimate monetized benefit obtained are deterministic. The remaining parameters are related to subjective perceptions, calculated using foreground values.  Table 2 shows the payoff matrix of the bidding collusion evolution game.

### 2.4. Model Solution

The steps for solving the model are shown in Figure 2.

According to Table 1, the prospective expectations and mean expectations for the bidders' sector to adopt the “engage in collusion” and “do not engage in collusion” strategies are

(4) $$\begin{array}{c} E_{11}=y*z*m*\left(V\left(F\right)+\alpha *R_{1}-\beta *V\left(S_{1}\right)\right)+\left(1-y\right)*z*m*\left(V\left(F\right)+\alpha *R_{1}-\beta *V\left(S_{1}\right)\right)+\\ y*\left(1-z\right)*m*\left(V\left(F\right)+\alpha *R_{1}-\beta *V\left(S_{1}\right)\right)+y*z*\left(1-m\right)*\left(V\left(F\right)+\alpha *R_{1}-\beta *V\left(S_{1}\right)\right)+\\ \left(1-y\right)*\left(1-z\right)*m*\left(V\left(F\right)+\alpha *R_{1}-\beta *V\left(S_{1}\right)\right)+y*\left(1-z\right)*\left(1-m\right)*\left(V\left(F\right)+\alpha *R_{1}-\beta *V\left(S_{1}\right)\right)\\ +\left(1-y\right)*\left(1-z\right)*\left(1-m\right)*\left(V\left(F\right)+\alpha *R_{1}-\beta *V\left(S_{1}\right)\right),\\ E_{12}=y*z*m*\left(V\left(F\right)+V\left(F_{2}\right)\right)+\left(1-y\right)*z*m*\left(V\left(F\right)+V\left(F_{2}\right)\right)+\\ y*\left(1-z\right)*m*\left(V\left(F\right)+V\left(F_{2}\right)\right)+y*z*\left(1-m\right)*\left(V\left(F\right)+V\left(F_{2}\right)\right)+\left(1-y\right)*\left(1-z\right)*m*\left(V\left(F\right)+V\left(F_{2}\right)\right)\\ +y*\left(1-z\right)*\left(1-m\right)*\left(V\left(F\right)+V\left(F_{2}\right)\right),\\ {\bar{E}}_{13}=x*E_{12}-\left(1-x\right)*E_{12}. \end{array}$$

The prospective expectations and mean expectations of firms with a high willingness to collude for “active collusion” and “inactive collusion” strategies are

(5) $$\begin{array}{c} E_{21}=x*z*m*\left(E*\text{SS}*V\left(F_{3}\right)-S_{3}-\beta *S_{4}+S_{2}\right)+\left(1-x\right)*z*m*\left(E*\text{SS}*\left(V\left(F_{3}\right)-S_{3}-\beta *S_{4}\right)+\right.\\ x*\left(1-z\right)*m*\left(E*\text{SS}*\left(V\left(F_{3}\right)-S_{3}-\beta *S_{4}+S_{2}\right)\right.+x*z*\left(1-m\right)*\left(E*\text{SS}*V\left(F_{3}\right)-S_{3}-\beta *S_{4}+S_{2}\right)\\ +\left(1-x\right)*\left(1-z\right)*m*\left(E*\text{SS}*V\left(F_{3}\right)-S_{3}-\beta *S_{4}+S_{2}\right)+\\ \left(1-x\right)*z*\left(1-m\right)*\left(E*\text{SS}*V\left(F_{3}\right)-S_{3}-\beta *S_{4}+S_{2}\right)+\\ \left(1-x\right)*\left(1-z\right)*\left(1-m\right)*\left(E*\text{SS}*V\left(F_{3}\right)-S_{3}-\beta *S_{4}+S_{2}\right),\\ E_{22}=x*z*m*\left(R_{3}*S_{2}+S_{5}\right)+\left(1-x\right)*z*m*\left(R_{3}*S_{2}+S_{5}\right)+x*\left(1-z\right)*m*\left(R_{3}*S_{2}+S_{5}\right)\\ +x*z*\left(1-m\right)*\left(R_{3}*S_{2}+S_{5}\right)+\left(1-x\right)*\left(1-z\right)*m*\left(R_{3}*S_{2}+S_{5}\right)\\ +\left(1-x\right)*z*\left(1-m\right)*\left(R_{3}*S_{2}+S_{5}\right)+x*\left(1-z\right)*\left(1-m\right)*\left(R_{3}*S_{2}+S_{5}\right),\\ {\bar{E}}_{23}=y*E_{21}-\left(1-y\right)*E_{22}. \end{array}$$

The prospective expectations and mean expectations of firms with low collusion intentions adopting the “report collusion” and “do not report collusion” strategies are

(6) $$\begin{array}{c} E_{31}=x*y*m*\left(V\left(F_{4}\right)-D*S_{6}\right)+\left(1-x\right)*y*m*\left(V\left(F_{4}\right)-D*S_{6}\right)+\\ x*\left(1-y\right)*m*\left(V\left(F_{4}\right)-D*S_{6}\right)+x*y*\left(1-m\right)*\left(V\left(F_{4}\right)-D*S_{6}\right)+\left(1-x\right)*\left(1-y\right)*m*F_{5}\\ +\left(1-x\right)*y*\left(1-m\right)*\left(V\left(F_{4}\right)-D*S_{6}\right)+\left(1-y\right)*\left(1-m\right)*\left(V\left(F_{4}\right)-D*S_{6}\right)\\ +\left(1-x\right)*\left(1-y\right)*\left(1-m\right)*\left(V\left(F_{4}\right)-D*S_{6}\right),\\ E_{32}=x*y*m*F_{5}+\left(1-x\right)*y*m*F_{5}+x*\left(1-y\right)*m*F_{5}+x*z*\left(1-m\right)*F_{5}\\ +\left(1-x\right)*\left(1-y\right)*m*F_{5}+x*\left(1-y\right)*\left(1-m\right)*F_{5}+\left(1-x\right)*\left(1-y\right)*z*F_{5}+\\ \left(1-x\right)*\left(1-y\right)*\left(1-m\right)*F_{5},\\ {\bar{E}}_{33}=z*E_{31}-\left(1-z\right)*E_{32}. \end{array}$$

The regulators' prospective expectations and mean expectations for a “strong regulatory model” and a “weak regulatory model” strategy are

(7) $$\begin{array}{c} E_{41}=x*y*z*\left(F_{6}+V\left(F_{7}\right)-V\left(S_{6}\right)\right)+\left(1-x\right)*y*z*\left(F6+V\left(F_{7}\right)-V\left(S_{6}\right)\right)+\\ x*\left(1-y\right)*z*\left(F_{6}+V\left(F_{7}\right)-V\left(S_{6}\right)\right)+x*y*\left(1-z\right)*\left(F_{6}+V\left(F_{7}\right)-V\left(S_{6}\right)\right)\\ +\left(1-x\right)*\left(1-y\right)*z*\left(F_{6}+V\left(F_{7}\right)-V\left(S_{6}\right)\right)+\\ \left(1-x\right)*y*\left(1-z\right)*\left(F_{6}+V\left(F_{7}\right)-V\left(S_{6}\right)\right)\\ +x*\left(1-y\right)*\left(1-z\right)*\left(F_{6}+V\left(F_{7}\right)-V\left(S_{6}\right)\right)+\\ \left(1-x\right)*\left(1-y\right)*\left(1-z\right)*\left(F_{6}+V\left(F_{7}\right)-V\left(S_{6}\right)\right),\\ E_{42}=x*y*z*\left(F_{6}+V\left(F_{7}\right)-V\left(S_{6}\right)+G*V\left(F_{7}\right)-D*V\left(S_{7}\right)+\right.\\ \left(1-x\right)*y*z*\left(F_{6}+V\left(F_{7}\right)-V\left(S_{6}\right)+G*V\left(F_{7}\right)-D*V\left(S_{7}\right)\right.\\ +x*\left(1-y\right)*z*F_{6}+x*\text{y}*\left(1-z\right)*\left(F_{6}+V\left(F_{7}\right)-V\left(S_{6}\right)+G*V\left(F_{7}\right)-D*V\left(S_{7}\right)\right.\\ +\left(1-x\right)*\left(1-y\right)*z*\left(F_{6}+V\left(F_{7}\right)-V\left(S_{6}\right)+G*V\left(F_{7}\right)-D*V\left(S_{7}\right)\right.\\ +\left(1-x\right)*y*\left(1-z\right)*\left(F6+V\left(F_{7}\right)-V\left(S_{6}\right)+G*V\left(F_{7}\right)-D*V\left(S_{7}\right)+\right.\\ x*\left(1-y\right)*\left(1-z\right)*\left(F_{6}+V\left(F_{7}\right)-V\left(S_{6}\right)+G*V\left(F_{7}\right)-D*V\left(S_{7}\right)\right.\\ +\left(1-x\right)*\left(1-y\right)*\left(1-z\right)*\left(F_{6}+V\left(F_{7}\right)-V\left(S_{6}\right)+G*V\left(F_{7}\right)-D*V\left(S_{7}\right)\right.,\\ {\bar{E}}_{43}=m*E_{41}-\left(1-m\right)*E_{42}. \end{array}$$

The replicated dynamic differential equation for the choice of an active strategy by bidders, high collusion willing firms, low collusion willing firms, and regulators can be expressed as

(8) $$\begin{array}{c} F\left(X\right)=\frac{\text{d}x}{\text{d}t}=x*\left(E_{11}-{\bar{E}}_{13}\right)=x*\left(1-x\right)*\left(E_{11}+E_{12}\right)=\\ x*\left(1-x\right)*\left(y*z*m\left(2V\left(F\right)+\alpha R_{1}+V\left(F_{2}\right)-\beta V\left(S_{1}\right)\right)+\left(1-z\right)*\left(2V\left(F\right)+\alpha R_{1}+V\left(F_{2}\right)-\beta V\left(S_{1}\right)\right)\right.\\ +z*m*\left(2V\left(F\right)+\alpha R_{1}+V\left(F_{2}\right)-\beta V\left(S_{1}\right)\right)+y*z*\left(2V\left(F\right)+\alpha R_{1}+V\left(F_{2}\right)-\beta V\left(S_{1}\right)\right)\left(\right),\\ F\left(Y\right)=\frac{\text{d}y}{\text{d}t}=y*\left(E_{21}-{\bar{E}}_{23}\right)=y*\left(1-y\right)*\left(E_{21}+E_{22}\right)=\\ =y*\left(1-y\right)*\left(z*x*m*\left(E*\text{SS}*V\left(F_{3}\right)-S_{3}-\beta *S_{4}+S_{2}+R_{3}*S_{2}+S_{5}-S_{2}\right)\right.\\ +\left(1-z\right)*\left(E*\text{SS}*V\left(F_{3}\right)-S_{3}-\beta *S_{4}+S_{2}+R_{3}*S_{2}+S_{5}-S_{2}\right)\\ +z*m*\left(\text{SS}*V\left(F_{3}\right)-S_{3}-\beta *S_{4}+S_{2}+R_{3}*S_{2}+S_{5}\right)\\ +x*z*\left(\text{SS}*V\left(F_{3}\right)-S_{3}-\beta *S_{4}+S_{2}+R_{3}*S_{2}+S_{5}\right),\\ F\left(Z\right)=\frac{\text{d}z}{\text{d}t}=z*\left(E_{31}-{\bar{E}}_{33}\right)=z*\left(1-z\right)*\left(E_{31}+E_{32}\right)=\\ =z*\left(1-z\right)*\left(x*y*m*\left(V\left(F_{4}\right)-D*V\left(S_{6}\right)+F_{5}\right)+\left(1-y\right)*\left(V\left(F_{4}\right)-D*V\left(S_{6}\right)+F_{5}\right)\right.\\ +\left(1-y\right)*m*\left(V\left(F_{4}\right)-D*V\left(S_{6}\right)+F_{5}\right)+x*y*\left(V\left(F_{4}\right)-D*V\left(S_{6}\right)+F_{5}\right),\\ F\left(M\right)=\frac{\text{d}m}{\text{d}t}=m*\left(E_{41}-{\bar{E}}_{43}\right)=m*\left(1-m\right)*\left(E_{41}+E_{42}\right)=\\ =m*\left(1-m\right)*\left(x*y*z*\left(2F_{6}+2V\left(F_{7}\right)-V\left(S_{6}\right)+G*V\left(F_{7}\right)-D*S_{7}\right)\right.\\ +\left(1-y\right)*\left(2F_{6}+2V\left(F_{7}\right)-V\left(S_{6}\right)+G*V\left(F_{7}\right)-D*S_{7}\right)\\ +y*z*\left(2F_{6}+2V\left(F_{7}\right)-V\left(S_{6}\right)+G*V\left(F_{7}\right)-D*S_{7}\right)\\ +x*y*\left(2F_{6}+2V\left(F_{7}\right)-V\left(S_{6}\right)+G*V\left(F_{7}\right)-D*S_{7}\right). \end{array}$$

When the government party's probability of engaging in collusion is 1, the government party receives a base benefit of *F*. The prospective value of *F* is

(9) $$\begin{array}{c} V\left(F\right)=\pi \left(1\right)*V\left(F\right)=F^{\theta }. \end{array}$$

When collusion is discovered, a loss of *S*_1_ is obtained, and the prospective value of *S*_1_ is

(10) $$\begin{array}{c} V\left(S_{1}\right)=\pi \left(1\right)*V\left(-S_{1}\right)=-\lambda S_{1}^{\theta }. \end{array}$$

Similarly, the foreground values of F2, F3, F4, S6, and F7 can be obtained.

The positive strategy dynamic game equation of quadrilateral game can be obtained by substituting the prospect value:

(11) $$\begin{array}{c} F\left(X\right)=\frac{\text{d}x}{\text{d}t}=x*\left(E_{11}-{\bar{E}}_{13}\right)=x*\left(1-x\right)*\left(E_{11}+E_{12}\right)\\ =x*\left(1-x\right)*\left(y*z*m\left(2F^{\theta }+\alpha R_{1}+F_{2}^{\theta }+\lambda \beta S_{1}^{\theta }\right)+\left(1-z\right)*\left(2F^{\theta }+\alpha R_{1}+F_{2}^{\theta }+\lambda \beta S_{1}^{\theta }\right)+\right.\\ z*m*\left(2F^{\theta }+\alpha R_{1}+F_{2}^{\theta }+\lambda \beta S_{1}^{\theta }\right)+y*z*\left(2F^{\theta }+\alpha R_{1}+F_{2}^{\theta }+\lambda \beta S_{1}^{\theta }\right)\left(\right),\\ F\left(Y\right)=\frac{\text{d}y}{\text{d}t}=y*\left(E_{21}-{\bar{E}}_{23}\right)=y*\left(1-y\right)*\left(E_{21}+E_{22}\right)=\\ =y*\left(1-y\right)*\left(z*x*m*\left(E*\text{SS}*F_{3}^{\theta }-S_{3}-\beta *S_{4}+S_{2}+R_{3}*S_{2}+S_{5}-S_{2}\right)+\right.\\ +\left(1-z\right)*\left(E*\text{SS}*F_{3}^{\theta }-S_{3}-\beta *S_{4}+S_{2}+R_{3}*S_{2}+S_{5}-S_{2}\right)\\ +z*m*\left(\text{SS}*F_{3}^{\theta }-S_{3}-\beta *S_{4}+S_{2}+R_{3}*S_{2}+S_{5}\right)+x*z*\left(\text{SS}*F_{3}^{\theta }-S_{3}-\beta *S_{4}+S_{2}+R_{3}*S_{2}+S_{5}\right),\\ F\left(Z\right)=\frac{\text{d}z}{\text{d}t}=z*\left(E_{31}-{\bar{E}}_{33}\right)=z*\left(1-z\right)*\left(E_{31}+E_{32}\right)=\\ =z*\left(1-z\right)*\left(x*y*m*\left(F_{4}^{\theta }+\lambda \;D*S_{6}^{\theta }+F5\right)+\left(1-y\right)*\left(F_{4}^{\theta }+\lambda \;D*S_{6}^{\theta }+F_{5}\right)\right.\\ +\left(1-y\right)*m*\left(F_{4}^{\theta }+\lambda \;D*S_{6}^{\theta }+F_{5}\right)+x*y*\left(F_{4}^{\theta }+\lambda \;D*S_{6}^{\theta }+F_{5}\right),\\ F\left(M\right)=\frac{\text{d}m}{\text{d}t}=m*\left(E_{41}-{\overset{\text{\_}}{E}}_{43}\right)=m*\left(1-m\right)*\left(E_{41}+E_{42}\right)=\\ =m*\left(1-m\right)*\left(x*y*z*\left(2F_{6}+2F_{7}^{\theta }+\lambda S_{6}^{\theta }+G*F_{7}^{\theta }-D*S_{7}\right)\right.\\ +\left(1-y\right)*\left(2F_{6}+2F_{7}^{\theta }+\lambda S_{6}^{\theta }-D*S_{7}\right)\\ +y*z*\left(2F_{6}+2F_{7}^{\theta }+\lambda S_{6}^{\theta }+G*F_{7}^{\theta }-D*S_{7}\right)+x*y*\left(2F_{6}+2F_{7}^{\theta }+\lambda S_{6}^{\theta }+G*F_{7}^{\theta }-D*S_{7}\right). \end{array}$$

## 3. Equilibrium Analysis of the Four-Party Game in Transportation Infrastructure Project Operation

### 3.1. Game Player Unilateral Stability Strategy

#### 3.1.1. Analysis of the Tenderer's Strategic Stability

Let *F*(*X*) = 0 and solve for *x* = 0, *x* = 1, *y* =  (*z* − 1) − *z∗m*/*z∗*(*m*+1)=*Y*^*∗*^. It follows from the stability theorem for replicating dynamic differential equations that *F*(*y*) = 0, ∂*F*(*x*)/∂*x* < 0, *x* is an evolutionary stabilization strategy.Since the range of values of *z*, *m* is [0, 1], in this article *Y*∗≤0.Thus, there are only two cases, *y* = *Y*∗ and *y* > *Y*∗.

When *y* = *Y*∗, F(*X*) = 0 is constantly established, and the stability point is *x* = 0, *x* = 1. Any value of *x* is a steady-state, i.e., the strategy of the construction unit does not change over time.

When *y* > *Y*∗, F(*X*) = 0 is constantly established, and $\left\{\begin{array}{c} \partial F\left(x\right)/\partial x>0,x\;=\;0\\ \partial F\left(x\right)/\partial x<0,x\;=\;1 \end{array}\right)$ is established. The stability point is *y* = 0, and any value of *x* is steady-state, indicating that the perceived costs of the positive pole strategy outweigh the benefits for the bidders, who prefer to bear the penalty of uncertainty rather than investing more.

The bidders' replicated dynamic phase diagram is shown in Figure 3.

#### 3.1.2. Analysis of the Progressive Stability of Firms with a High Willingness to Collude

Let *F*(*Y*) = 0 and solve for *y* = 0, *y* = 1,

(12) $$\begin{array}{c} z=-\frac{E*\text{SS}*F_{3}^{\theta }-S_{3}-\beta *S_{4}+S_{2}+R_{3}*S_{2}+S_{5}-S_{2}}{\begin{array}{c} x*m*\left(E*\text{SS}*F_{3}^{\theta }-S_{3}-\beta *S_{4}+S_{2}+R_{3}*S_{2}+S_{5}-S_{2}\right)-\left(E*\text{SS}*F_{3}^{\theta }-S_{3}-\beta *S_{4}+S_{2}+R_{3}*S_{2}+S_{5}-S_{2}\right)+\\ m*\left(\text{SS}*V\left(F_{3}\right)-S_{3}-\beta *S_{4}+S_{2}+R_{3}*S_{2}+S_{5}\right)+x*\left(\text{SS}*F_{3}^{\theta }-S_{3}-\beta *S_{4}+S_{2}+R_{3}*S_{2}+S_{5}\right) \end{array}}=Z^{*}. \end{array}$$

It follows from the stability theorem for replicating dynamic differential equations that *F*(*y*) = 0, ∂*F*(*y*)/∂*y* < 0, x is an evolutionary stabilization strategy.

When *z* = *Z*∗, *F*(*y*) = 0 is constantly established. The stability point is *y* = 0, *y* = 1, and any value of *y* is steady-state. The high collusion unit's strategy does not change over time.

When *z* < *Z*∗, *F*(*y*) = 0 is constantly established, and $\left\{\begin{array}{c} \partial F\left(y\right)/\partial y>0,y\;=\;0\\ \partial F\left(y\right)/\partial y<0,y\;=\;1 \end{array}\right)$ is established. The stability point is *y* = 1, and any value of *x* is steady-state. This suggests that parties with a high willingness to collude perceive the benefits of an aggressive strategy outweigh the costs. The benefits include a variety of gains. As shown by prospect theory, game subjects are usually reluctant to take losses when faced with gains, and parties with a high willingness to collude tend to adopt collusive strategies.

When *z* > *Z*∗, *F*(*y*) = 0 is constantly established, and $\left\{\begin{array}{c} \partial F\left(y\right)/\partial y>0,y\;=\;0\\ \partial F\left(y\right)/\partial y<0,y\;=\;1 \end{array}\right)$ is established. The stability point is *y* = 0, and any value of *x* is steady-state, indicating that the penalties and losses received by the building operator in providing low-quality services are less than the gains under this strategy. In this case, the building operator tends to choose a speculative strategy to obtain higher returns. The party willing to collude replicates the dynamic phase diagram, as shown in Figure 4.

#### 3.1.3. Analysis of the Progressive Stability of Firms with a Low Willingness to Collude

Let *F*(*Z*) = 0 and solve for *z* = 0, *z* = 1, *m* =  *λY*_1_^*θ*^ − *λY*_2_^*θ*^+*y*/*y* − 1  = M^∗^. It follows from the stability theorem for replicating dynamic differential equations that F(*z*) = 0, ∂*F*(*z*)/∂*z* < 0, *z* is an evolutionary stabilization strategy.

When *m* = *M*∗, *F*(*Z*) = 0 is constantly established. The stability point is *z* = 0, *z* = 1, and any value of *z* is steady-state. The strategy of the low collusion unit does not change over time.

When *m* < *M*∗, *F*(*Z*) = 0 is constantly established, and $\left\{\begin{array}{c} \partial F\left(z\right)/\partial z>0,z\;=\;0\\ \partial F\left(z\right)/\partial z\;<0,z\;=\;1 \end{array}\right)$ is established. The stability point is *z* = 1, and any value of *z* is steady-state, suggesting that, for the low colluder, the perceived benefits of adopting an aggressive strategy outweigh the costs. In this case, the low colluding party tends to adopt a strategy of reporting the collusion.

When *z* > *Z*∗, *F*(*Z*) = 0 is constantly established, and $\left\{\begin{array}{c} \partial F\left(z\right)/\partial z>0,z\;=\;0\\ \partial F\left(z\right)/\partial z<0,z\;=\;1 \end{array}\right)$ is established. The stability point is *z* = 0, and any value of *z* is steady-state, suggesting that users have greater benefits from adopting nonreporting collusion. The low collusion willingness side tends to be associated with a nonreporting strategy. The low collusion willingness side replicates the dynamic phase diagram, as shown in Figure 5.

#### 3.1.4. Progressive Stability Analysis of Regulators

Let *F*(*M*) = 0 and solve for *m* = 0, *m* = 1, *x* =  (*y* − 1+*yz* − ((1 − *y*)*G∗F*_7_^*θ*^)/(2*F*_6_+2*F*_7_+*λS*_6_+*G∗F*_7_ − *D∗S*_7_)/(*yz*+*y*))  = *X*^∗^. It follows from the stability theorem for replicating dynamic differential equations that F(m) = 0, ∂*F*(*m*)/∂*m* < 0, *m* is an evolutionary stabilization strategy.

When *x* = *X*∗, *F*(*M*) = 0 is constantly established. The stability point is *m* = 0, *m* = 1, and any value of *m* is steady-state. The strategy of the low collusion unit does not change over time.

When *x* < *X*∗, *F*(*M*) = 0 is constantly established, and $\left\{\begin{array}{c} \partial F\left(m\right)/\partial m>0,m\;=\;0\\ \partial F\left(m\right)/\partial m<0,m\;=\;1 \end{array}\right)$ is established. The stability point is *m* = 1, and any value of *m* is steady-state, suggesting that the supervisory authority's perceived benefits outweigh the costs of an active strategy. In such cases, regulators tend to adopt strong regulatory measures against collusive behavior.

When *x* > *X*∗, *F*(*M*) = 0 is constantly established, and $\left\{\begin{array}{c} \partial F\left(m\right)/\partial m>0,m\;=\;0\\ \partial F\left(m\right)/\partial m<0,m\;=\;1 \end{array}\right)$ is established. The stability point is *m* = 0, and any value of *m* is a steady-state, suggesting a greater gain for the regulators in adopting a weak regulatory strategy. In this case, there is a greater probability that the regulators will forgo regulation and choose not to regulate collusion. See Figure 6 for a phase diagram of regulator replication dynamics.

### 3.2. Strategy Portfolio Stability Analysis

Let F(*x*) = *F*(*y*) = F(*z*) = F(m) = 0. The equilibrium points can be obtained as follows: *E*_1_(0,0,0,0), *E*_2_(1,0,0,0), *E*_3_(0,1,0,0), *E*_4_(0,0,1,0), *E*_5_(0,0,0,1), *E*_6_(1,1,0,0), *E*_7_(1,0,1,0), *E*_8_(1,0,0,1), *E*_9_(0,1,1,0), *E*_10_(0,1,0,1), *E*_11_(0,0,1,1), *E*_12_(1,1,1,0), *E*_13_(1,1,0,1), *E*_14_(1,0,1,1), *E*_15_(0,1,1,1), *E*_16_(1,1,1,1), *E*_17_(*x*^*∗*^, *y*^*∗*^, *z*^*∗*^, *m*^*∗*^); *E*_17_ is the mixed strategy equilibrium point. Suppose the equilibrium point in the three-way evolutionary game is ESS. In that case, it must be satisfied that the equilibrium point is a pure strategy equilibrium, and therefore only the asymptotic stability of *E*_1_ to *E*_16_ needs to be discussed. The asymptotic stability of the system can be obtained from the analysis of the Jacobian matrix, as proposed by Friedman:

(13) $$\begin{array}{c} J=\left[\begin{array}{cccc} \frac{\partial F\left(x\right)}{\partial x} & \frac{\partial F\left(x\right)}{\partial y} & \frac{\partial F\left(x\right)}{\partial z} & \frac{\partial F\left(x\right)}{\partial m}\\ \frac{\partial F\left(y\right)}{\partial x} & \frac{\partial F\left(y\right)}{\partial y} & \frac{\partial F\left(y\right)}{\partial z} & \frac{\partial F\left(y\right)}{\partial m}\\ \frac{\partial F\left(z\right)}{\partial x} & \frac{\partial F\left(z\right)}{\partial y} & \frac{\partial F\left(z\right)}{\partial z} & \frac{\partial F\left(z\right)}{\partial m}\\ \frac{\partial F\left(m\right)}{\partial x} & \frac{\partial F\left(m\right)}{\partial y} & \frac{\partial F\left(m\right)}{\partial z} & \frac{\partial F\left(m\right)}{\partial m} \end{array}\right]. \end{array}$$

Each of the 16 equilibrium points is substituted into the Jacobian matrix. If the eigenvalues of the corresponding matrix are all negative, the equilibrium point is the system's ESS. The stability of each point is shown in Table 3.

The calculations reveal that this article should analyze the game's stabilization strategy in two scenarios.

Scenario 1: for all parties, the benefits of collusion are greater than the potential costs. In this case, *M*_2_, *M*_3_, *M*_5,_ and *M*_6_ are all greater than 0. In the game process, the benefits of the collusion process are greater than the costs incurred by the bidding parties, including direct costs, reputational losses, and potential expansion. In this case, the table shows that *E*_16_(1,1,1,1) is the equilibrium point, and that the evolving equilibrium strategies are: engage in collusion, active participation in the collusion, report the collusion, weak regulatory model.

Scenario 2: the benefits of collusion are less than the potential costs for all parties. In this scenario, *M*_2_, *M*_3_, *M*_5,_ and *M*_6_ are all less than 0. In the game, the benefits of collusion to the bidding parties are greater than their costs, including direct costs, reputational damage, and potential expansion.  Table 4 shows that there is no stable equilibrium in this case.

## 4. Analysis of Simulations

### 4.1. Initial Parameters Setting

The model is assigned according to the real situation, and numerical simulation is carried out using Matlab 2020b. These choices intuitively demonstrate the influence of key factors on the evolutionary process and results of the multiparty game in the government project bidding process and verify the validity of the evolutionary stability analysis. The studied behavior is vertical collusion in the bidding process of government investment projects. As such, all parties are bound by relevant laws and regulations and hidden costs, and they tend to choose negative strategies at the beginning of the period. The probability of choosing positive strategies is less than 0.5. The probability of choosing the positive strategy is even lower due to the fear of loss and retaliation for reporting vertical collusion. According to the actual situation and this paper's assumptions, *x*, y, *z*, and *m* are set as 0.4, 0.3, 0.2, and 0.3, respectively, see Table 5.

### 4.2. Single-Factor Sensitivity Analysis

#### 4.2.1. Impact of Changes in the Social Benefits of Project Completion Base

When *F* = {12,18,24,30}, the process and results of the evolution of the thematic strategy of the quadratic game are shown in Figure 7.

As seen in Figure 6, the increase in project completion benefits as the bidders collude impacts each of the four-party's evolutionary strategies. The more obvious change is for the bidders. With the increase of the social base gain, the probability of the bidders to adopt the collusion strategy shows an increase in the magnitude of the change, and the speed of evolution to a stable strategy becomes faster. However, the reduction of social base revenue can only reduce the occurrence of collusion in the short term and delay the evolution to a stable point. Still, it cannot control the occurrence of collusion.

#### 4.2.2. Impact of Changes in Risk Attitude Factor

When *θ* = {0.8, 0.5, 0.3, 0.2}, the process and results of the evolution of the thematic strategy of the quadratic game are shown in Figure 8.

As shown in Figure 8, as the risk attitude increases, the probability of choosing collusion-related strategies decreases for each project participant. In the four-party game, with the change of risk attitude, the strategy change is more evident in the evolution trend of the bidding party and the party with high collusion willingness. As the risk attitude decreases, we find that the remaining conditions are unchanged. The initial degree of influence regarding the change in risk attitude on the parties' choice is greater than the social base gain. However, the change in risk attitude does not change each group's final choice. Only at the initial stage can the probability of collusive behavior be reduced between the bidding party and the party with high collusion willingness.

#### 4.2.3. Impact of Changes in the Level of Competition in the Market

When SS = {0.5, 0.75, 1,1.25}, the process and results of the evolution of the thematic strategy of the quadratic game are shown in Figure 9.

As shown in Figure 9, the initial probability of bidders and parties with a high willingness to collude to choose collusion strategies also decreases as the degree of market competition continues to decline. However, the tenderers' willingness to collude decreases less in the initial period when the degree of market competition decreases. It decreases more sharply only after maintaining a smaller degree of market competition. However, a decrease in the degree of market competition does not affect each participant's final evolutionary outcome.

#### 4.2.4. Impact of Changes in the Probability of Collusion Being Detected

When *β* = *D* ={0.8, 0.5, 0.3, 0.2}, the process and results of the evolution of the thematic strategy of the quadratic game are shown in Figure 10.

As shown in Figure 10, as the probability of detecting collusion rises, the probability that the high collusion willing party and the tenderer will choose the collusion strategy decreases to some extent. Still, the high collusion willing party is more sensitive to the probability of collusion being detected. At the same time, as the probability of collusion detection being reported decreases, the probability of low collusion willing parties choosing to collude also decreases. Therefore, in controlling vertical collusion, it is essential to establish smooth reporting channels, protect the privacy of those who report violations, and avoid retaliation against whistleblowers. At the same time, it is important to increase supervision and establish a regular inspection and monitoring mechanism. The establishment of an effective monitoring system will improve the effectiveness of controls on collusion.

### 4.3. Impact of Internal Oversight Measures on Vertical Collusion

To further investigate the influence of the internal supervision mechanism in government projects' bidding process, the simulation analysis was conducted by setting *z* = 0 and *z* = 0.9 to indicate the two states of the low collusion tendency group to report or not to report collusion. The evolution process of different initial strategies was simulated for three parties, tenderers, high collusion willing parties, and supervisory agencies, and the results are shown in Figure 11.

From Figure 11, when *z* = 0, i.e., when low collusion-prone firms choose to engage in collusion without reporting, the stabilization strategy of the remaining participants in the bidding process is not unique due to the influence of many external factors. When *z* = 0.9, it has a unique stabilization evolution strategy (participation in collusion, active collusion, and strong regulatory model). Therefore, low collusion-prone firms are encouraged to report collusion; strengthening internal supervision has a better effect on the control of collusion.

### 4.4. The Impact of External Punishment Mechanisms

The evolutionary strategy's impact was analyzed by setting the change in the punishment and supervision cost level when collusion was detected to investigate the effectiveness and feasibility of the external punishment mechanism in controlling collusion. Simulations were conducted to analyze the evolutionary process of different initial strategies of the three parties: the tenderer, the party with high willingness to collude, and the party with low willingness to collude. The results are shown in Figure 12.

As shown in Figure 12, as external penalties increase, the benefits gained by choosing to collude shift from higher than losses (low penalties) to medium penalties (the benefits of choosing to collude are equal to the losses when punished) and high penalties (the benefits of choosing to collude are lower than the losses when discovered). The probability of firms with higher willingness to collude engaging in collusion gradually decreases; however, as the cost of supervision increases, the probability of regulators adopting weak supervision also increases. Therefore, while increasing the intensity of control, attention should be paid to the equilibrium conditions. Such attention can avoid a decrease in the supervisory body's willingness to supervise due to an excessive increase in external penalties.

## 5. Conclusions

This study focuses on the generation and control of collusion in the bidding process of government projects in China. It examines how to improve the quality of control of bidding collusion by considering different groups of enterprises and society's external supervision mechanism. The findings revealed the following.

1. Establishing an effective external supervision mechanism and social supervision system can effectively reduce the probability of collusion among all participants and achieve the quality of control over speculative behavior in the bidding process. The quality of the supervision system is closely related to the interests of the supervisory body, the benefits of reporting illegal behavior by social groups, and whether the report will bring retaliation from the tenderer and the colluding enterprises. In the control process, it is first necessary to reduce the cost of supervision and increase the incentives for supervisory bodies. Additionally, the application of deep learning, artificial intelligence, and other technologies should be vigorously promoted in the bidding process. Furthermore, a control mechanism should be established, combining artificial intelligence technology and manual auditing to reduce control costs.
2. While establishing an effective regulatory mechanism, the reward and punishment mechanism should be improved to increase the punishment for law violations. Punishments can be imposed in the form of restrictions on bidding, social publicity, fines, and reduction of qualifications to increase the risk awareness of all participants in bidding and discourage those with a higher willingness to collude from participating in collusive behavior. At the same time, regular “look-back” inspections of phased government bidding projects should be carried out, with each region cross-checking the project's compliance to avoid concealment in the monitoring process.
3. The bidding threshold and profitability of government bidding projects should be gradually raised under reasonable conditions. The level of competition in the market for government bidding projects should be reduced to control the willingness of project collusion participants. The simulation results show that the willingness of all parties to collude is low when the market is less competitive. Therefore, reasonably controlling the threshold and profitability of government projects can better control collusion. This will facilitate compliance and healthy operation of government bidding projects and the overall bidding market.
4. Through research, we found that simply increasing the fines for illegal acts or improving the supervision cannot completely solve the vertical collusion in the bidding process of government investment projects. In the actual control process, we need to focus on the combination of internal supervision and external supervision system to enhance the law-abiding consciousness of each interest body, so as to realize that each interest body is unwilling to collude in thought and dare not collude in action, and to promote the effective operation of the bidding market of government investment projects.

The limitations of this study are the following two points.

1. This study is based on the assumptions of non-fully rational economists and prospect theory. Still, in the government project bidding process, the decision of each game subject is influenced by random factors. Future research can examine the influence of random factors in the decision-making process and consider the influence of subjective emotions. Such an approach will make the results more in line with reality.
2. This study examines vertical collusion in government investment projects, and the scope is not broad enough; widespread horizontal collusion is not considered. Future research may consider adding horizontal collusion to enhance the scalability of the research results.

## Figures and Tables

**Figure 1:** Four-way diagram of the game.

**Figure 2:** Calculation logic table.

**Figure 3:** Tenderer replicates dynamic phase diagram.

**Figure 4:** High collusion replicates dynamic phase diagram.

**Figure 5:** Low collusion replicates dynamic phase diagram.

**Figure 6:** Regulators collusion replicates dynamic phase diagram.

**Figure 7:** (a) Impact of changes in the social benefits of project completion base on the evolution of the high tenderers' strategy. (b) Impact of changes in the social benefits of project completion base on the evolution of the high collusion's strategy. (c) Impact of changes in the social benefits of project completion base on the evolution of the low collusion's strategy. (d) Impact of changes in the social benefits of project completion based on the evolution of the regulator's strategy.

**Figure 8:** (a) Impact of changes in risk attitude coefficients on the evolution of the tenderers' strategies. (b) Impact of changes in risk attitude coefficients on the evolution of high collusion strategies. (c) Impact of changes in risk attitude coefficients on the evolution of low collusion strategies. (d) Impact of changes in risk attitude coefficients on the evolution of regulators' strategies.

**Figure 9:** (a) The impact of changing levels of market competition on the evolution of tenderers' strategies. (b) The impact of changing levels of market competition on the evolution of high collusion strategies. (c) The impact of changing levels of market competition on the evolution of low collusion strategies. (d) The impact of changing levels of market competition on the evolution of regulators' strategies.

**Figure 10:** (a) The impact of changing levels of market competition on the evolution of tenderers' strategies. (b) The impact of changing levels of market competition on the evolution of high collusion strategies. (c) The impact of changing levels of market competition on the evolution of low collusion strategies. (d) The impact of changing levels of market competition on the evolution of regulators' strategies.

**Figure 11:** (a) The impact of strong supervision by internal oversight mechanisms on quadrilateral games. (b) Impact of nonoversight by internal oversight bodies on the quadrilateral game.

**Figure 12:** (a) Impact of changes in external penalty mechanisms (initial situation). (b) Impact of changes in external penalty mechanisms (medium penalty levels). (c) Impact of changes in external penalty mechanisms (high penalty levels).

**Table 1:** Parameters and explanation.

Parameter	Explanation
*R*_1_	Risk of substandard capacity
*F*	Base earnings
*F*_3_	Scale-up incentive
*F*_5_	Nonreporting of collusive behavior gain
*F*_7_	Regulator collusion gain
*S*_2_	Winning bid gain
*S*_4_	Collusion discovery loss
*S*_6_	Losses from reported collusion being resisted
*E*	Probability of winning a bid by a firm with a high willingness to collude
*D*	Probability of detection of reported collusion
*β*	Probability of collusion being detected by the bidders
*λ*	Loss avoidance factor
*R*_3_	Probability of winning a bid
*F*_2_	Trust rising gain
*F*_4_	Recognition gain
*F*_6_	Regulatory gain
*S*_1_	Tenderer collusion discovery loss
*S*_3_	Collusion additional expense loss
*S*_5_	Reduced expansion loss
*S*_7_	Regulator collusion detected loss
SS	Degree of market competition
*G*	Probability of regulatory firms choosing to collude
*α*	Probability of colluding firms not meeting capacity standards
*θ*	Risk attitude coefficient

**Table 2:** Revenue matrix.

Strategy selection		Low collusion	Tenderers			
			Engage in collusion		Not engage in collusion	
			Active collusion	Inactive collusion	Active collusion	Inactive collusion
Regulators	Strong regulatory model	Reporting collusion	V(F)+*α*^*∗*^R_1_ − *β*^*∗*^V(S_1_)	V(F)+*α*^*∗*^R_1_ − *β*^*∗*^V(S_1_)	V(F)+F_2_	V(F)+V(F_2_)
			E^*∗*^SS^*∗*^(V(F_3_) − S_3_ − *β*^*∗*^*S*_4_+S_2_)	*R*_3_^*∗*^ *S*_2_+S_5_	E∗SS∗(V(F_3_) − S_3_-*β*^*∗*^S_4_)	*R*_3_^*∗*^ *S*_2_+S_5_
			V(F_4_) − D^*∗*^S_6_	V(F_4_) − D^*∗*^S_6_	V(F_4_) − D^*∗*^S_6_	V(F_4_) − D^*∗*^S_6_
			*F*_6_+V(F_7_) − V(S_6_)	*F*_6_+V(F_7_) − V(S_6_)	*F*_6_+V(F_7_) − V(S_6_)	*F*_6_+V(F_7_) − V(S_6_)
		Not reporting collusion	V(F)+*α*∗R_1_-*β*^*∗*^V(S_1_)	V(F)+*α*∗R_1_-*β*^*∗*^V(S_1_)	V(F)+V(F_2_)	V(F)+V(F_2_)
			E^*∗*^SS^*∗*^(V(F_3_) − S_3_ − *β*^*∗*^*S*_4_+S_2_)	*R*_3_^*∗*^ *S*_2_+S_5_	E∗SS∗(V(F_3_ − S_3_ − *β*∗S_4_)	*R*_3_^*∗*^ *S*_2_+S_5_
			*F*_5_	*F*_5_	*F*_5_	*F*_5_
			*F*_6_+V(F_7_) − V(S_6_)	*F*_6_+V(F_7_) − V(S_6_)	*F*_6_+V(F_7_) − V(S_6_)	*F*_6_+V(F_7_) − V(S_6_)
	Weak regulatory model	Reporting collusion	V(F)+*α*^*∗*^R_1_ − *β*^*∗*^V(S_1_)	V(F)+*α*∗R_1_ − *β*^*∗*^V(S_1_)	V(F)+V(F_2_)	V(F)+V(F_2_)
			E^*∗*^SS^*∗*^(V(F_3_) − S_3_ − *β*^*∗*^*S*_4_+S_2_)	*R*_3_^*∗*^ *S*_2_+S_5_	E^*∗*^SS^*∗*^(V(F_3_) − S_3_ − *β*∗S_4_)	*R*_3_^*∗*^ *S*_2_+S_5_
			V(F_4_) − D^*∗*^S_6_	V(F_4_) − D^*∗*^S_6_	V(F_4_) − D^*∗*^S_6_	V(F_4_) − D^*∗*^S_6_
			*F*_6_+V(F_7_) − V(S_6_)+G^*∗*^F_7_ − D∗S_7_	*F*_6_+V(F_7_) − V(S_6_)+G^*∗*^F_7_ − D^*∗*^S_7_	*F*_6_+V(F_7_) − V(S_6_)+G^*∗*^F_7_ − D^*∗*^S_7_	*F*_6_+V(F_7_) − V(S_6_)+G^*∗*^F_7_ − D^*∗*^S_7_
		Not reporting collusion	V(F)+*α*∗R_1_ − *β*^*∗*^V(S_1_)	V(F)+*α*∗R_1_ − *β*^*∗*^V(S_1_)	V(F)+V(F_2_)	V(F)+V(F_2_)
			E^*∗*^SS^*∗*^(V(F_3_) − S_3_ − *β*^*∗*^*S*_4_+S_2_)	*R*_3_^*∗*^ *S*_2_+S_5_	E^*∗*^SS^*∗*^(V(F_3_) − S_3_ − *β*^*∗*^S_4_)	*R*_3_^*∗*^ *S*_2_+S_5_
			F_5_	F_5_	F_5_	F_5_
			*F*_6_+V(F_7_) − V(S_6_)+G^*∗*^V(F_7_) − D^*∗*^S_7_	*F*_6_+V(F_7_) − V(S_6_)+G^*∗*^F_7_-D∗S_7_	*F*_6_+V(F_7_) − V(S_6_)+G^*∗*^V(F_7_)-D∗S_7_	*F*_6_+V(F_7_) − V(S_6_)+G^*∗*^V(F_7_) − D^*∗*^S_7_

**Table 3:** Eigenvalues.

Equalization points	Eigenvalue *λ*_1_	Eigenvalue *λ*_2_	Eigenvalue *λ*_3_	Eigenvalue *λ*_4_
*E*_1_(0,0,0,0)	*M*_1_	*M*_2_	*M*_4_	*M*_6_
*E*_2_(1,0,0,0)	−*M*_1_	*M*_2_	*M*_4_	*M*_6_
*E*_3_(0,1,0,0)	*M*_1_	−*M*_2_	0	0
*E*_4_(0,0,1,0)	0	0	−*M*_4_	*M*_6_
*E*_5_(0,0,0,1)	*M*_1_	*M*_2_	2*M*_4_	−M_6_
*E*_6_(1,1,0,0)	−*M*_1_	−*M*_2_	*M*_4_	*M*_5_
*E*_7_(1,0,1,0)	0	*M*_3_	−*M*_4_	*M*_6_
*E*_8_(1,0,0,1)	−M_1_	*M*_2_	2*M*_4_	−M_6_
*E*_9_(0,1,1,0)	*M*_1_	0	0	*M*_5_
*E*_10_(0,1,0,1)	*M*_1_	−*M*_2_	0	0
*E*_11_(0,0,1,1)	*M*_1_	*M*_3_	−2*M*_4_	−*M*_6_
*E*_12_(1,1,1,0)	−*M*_1_	−*M*_3_	−*M*_4_	3*M*_5_
*E*_13_(1,1,0,1)	−*M*_1_	−*M*_2_	2*M*_4_	−*M*_5_
*E*_14_(1,0,1,1)	−*M*_1_	*M*_2_ + 2*M*_3_	−2*M*_4_	−*M*_6_
*E*_15_(0,1,1,1)	3*M*_1_	−*M*_3_	0	−*M*_5_
*E*_16_(1,1,1,1)	−3*M*_1_	−M_2_−2*M*_3_	−2*M*_4_	−3*M*_5_

*M*_1_ = 2*F*^*θ*^+*αR*_1_+*F*_2_^*θ*^+*λβS*_1_^*θ*^; *M*_2_ = *E∗*SS*∗F*_3_^*θ*^ − *S*_3_ − *β∗S*_4_+*S*_2_+*R*_3_*∗S*_2_+*S*_5_ − *S*_2_; *M*_3_ = SS*∗F*_3_^*θ*^ − *S*_3_ − *β∗S*_4_+*S*_2_+*R*_3_*∗S*_2_+*S*_5_; *M*_4_ = *F*_4_^*θ*^+*λ*  *D∗S*_6_^*θ*^+*F*_5_; *M*_5_ = 2*F*_6_+2*F*_7_^*θ*^+*λS*_6_^*θ*^+*G∗F*_7_^*θ*^ − *D∗S*_7_; *M*_6_ = 2*F*_6_+2*F*_7_^*θ*^+*λS*_6_^*θ*^ − *D∗S*_7_.

**Table 4:** Stabilization table.

Equalization points	Scenario 1					Scenario 2				
	*λ*_1_	*λ*_2_	*λ*_3_	*λ*_4_	Stability	*λ*_1_	*λ*_2_	*λ*_3_	*λ*_4_	Stability
*E*_1_(0,0,0,0)	+	+	+	+	−	+	−	+	−	−
*E*_2_(1,0,0,0)	−	+	+	+	−	−	−	+	−	−
*E*_3_(0,1,0,0)	+	−	0	0	−	+	+	0	0	−
*E*_4_(0,0,1,0)	0	0	−	+	−	0	0	−	−	−
*E*_5_(0,0,0,1)	+	+	+	−	−	+	−	+	+	−
*E*_6_(1,1,0,0)	−	−	+	+	−	−	+	+	−	−
*E*_7_(1,0,1,0)	0	+	−	+	−	0	−	−	−	−
*E*_8_(1,0,0,1)	−	+	+	−	−	−	−	+	−	−
*E*_9_(0,1,1,0)	+	0	0	+	−	+	0	0	−	−
*E*_10_(0,1,0,1)	+	−	0	0	−	+	+	0	0	−
*E*_11_(0,0,1,1)	+	+	−	−	−	+	−	−	+	−
*E*_12_(1,1,1,0)	−	−	−	+	−	−	+	−	−	−
*E*_13_(1,1,0,1)	−	−	+	−	−	−	+	+	+	−
*E*_14_(1,0,1,1)	−	+	−	−	−	−	−	−	+	−
*E*_15_(0,1,1,1)	+	−	0	−	−	+	+	0	+	−
*E*_16_(1,1,1,1)	−	−	−	−	ESS	−	+	−	+	−

**Table 5:** Assignment table.

Parameters	Values
*R*_1_	−2
*F*	12
*F*_3_	2
*F*_5_	3
*F*_7_	1
*S*_2_	8
*S*_4_	2
*S*_6_	4
*E*	0.5
*D*	0.5
*β*	0.5
*λ*	0.5
*R*_3_	0.3
*F*_2_	8
*F*_4_	2
*F*_6_	6
*S*_1_	4
*S*_3_	5
*S*_5_	3
*S*_7_	2
SS	0.5
*G*	0.5
*α*	0.7
*θ*	0.5

## Data Availability

The raw data supporting the conclusions of this article will be made available by the authors, without undue reservation.
